# Clinical Efficacy of Tuomin Zhiti Decoction in Allergic Rhinitis

**DOI:** 10.1155/2022/8616075

**Published:** 2022-06-21

**Authors:** Jian-Xin Zhang, Wen-Yan Wang

**Affiliations:** Department of Oto-Rhino-Laryngology Head and Neck Surgery, Weihai Municipal Hospital, Weihai, Shandong, China

## Abstract

Allergic rhinitis (AR) is a noninfectious inflammatory disease seriously affecting the quality of life. This study aimed to assess the efficacy of the Tuomin Zhiti decoction in allergic rhinitis and to provide a reference for clinical treatment. One hundred patients with AR treated in the Department of Otolaryngology of our hospital from January 2019 to December 2020 were recruited and assigned via a random number table method (1 : 1) to receive either oral loratadine and mometasone nasal spray (control group) or the Tuomin Zhiti decoction plus oral loratadine and mometasone nasal spray (study group). The total clinical efficacy was 86% (43/50) in the study group, which was significantly higher than that of 64% (32/50) in the control group. After treatment, the Total Nasal Symptoms Scores (TNSS) and Rhinoconjunctivitis Quality of Life Questionnaire (RQLQ) scores between the two groups were similar, but 12 weeks after treatment, the study group had significantly lower TNSS and RQLQ scores than the control group. After treatment, the study group obtained lower levels of interleukin (IL)-4 and higher levels of interferon-*γ* (IFN-*γ*) than the control group. Significantly lower post-treatment peripheral blood eosinophil count (EOS) and eosinophil cationic protein (ECP) levels were observed in the study group in contrast to those of the control group. The Tuomin Zhiti decoction for the treatment of AR patients alleviates their clinical symptoms, reduces the inflammatory responses, enhances the immune function of patients by regulating IL-4 and IFN-*γ*, and lowers the long-term recurrence rate.

## 1. Introduction

Allergic rhinitis (AR) is a noninfectious inflammatory disease of the nasal mucosa caused by the release of mediators (mainly histamine) mediated primarily by IgE in atopic individuals after exposure to allergens, with the involvement of multiple immunoreactive cells and cytokines [1, 2]. It is a multifactorial disease closely related to genetics and allergen exposure, characterized by main symptoms such as paroxysmal sneezing, clear nasal discharge, nasal congestion, and nasal itching; hyposmia is infrequently found in some cases [3, 4]. The long duration of symptoms and the lengthy treatment period of AR drastically compromise the patients' quality of life. The treatment of AR primarily focuses on avoidance of allergen exposure, symptom relief, standardized immunotherapy, and health education, and with the popularization of new methods such as intranasal antihistamines and intranasal steroids, the symptoms of AR have been effectively controlled. However, issues such as poor compliance and high reoccurrence rate remain to be addressed [5, 6].

AR belongs to the category of “congested nose” in traditional Chinese medicine (TCM), which is associated with internal deficiencies of internal organs and healthy qi and external invasion of external evil qi. The pathogenesis of AR is closely correlated with the weakness of the spleen and stomach [7, 8]. The application of TCM in AR is yet to be popularized and is mostly empirical and randomized controlled studies on the application of TCM in AR are scarce. The Tuomin Zhiti decoction is a modified TCM formula by our academician Wang Qi, which is designed based on the idea of “key prescriptions for primary symptoms” to address the main issues concerning the pathogenesis of AR, namely, “the inherent poor physique and the external invasion of alien qi that triggers the heat in the nose and dries up the nasal orifices.” Its prescription focuses on the treatment of both the physique and the symptoms, with the efficacy of desensitizing and clearing heat, dispersing evil, and clearing orifices [9]. Herein, the Tuomin Zhiti decoction was used as an adjunctive treatment for AR patients, and the results are reported below.

## 2. Materials and Methods

### 2.1. General Information

This study was a prospective randomized controlled study with a single-blind (investigator) method. One hundred patients with allergic rhinitis (AR) treated in the Department of Otolaryngology of our hospital from January 2019 to December 2020 were recruited and divided into a control group and a study group using the random number table method, with 50 cases in each group. All subjects enrolled were informed about the process and purpose of the study and signed an informed consent form. The study was approved by the ethics committee of Weihai Municipal Hospital with the approval number of CC-2019/0134. The protocol followed the ethical principles of the Declaration of Helsinki [10].

### 2.2. Inclusion and Exclusion Criteria

#### 2.2.1. Inclusion Criteria

Patients who met the diagnostic criteria for moderate to severe persistent AR; who met the international diagnostic criteria for AR (ARIA) [11]: (a) clinical history symptoms: 2 or more symptoms of sneezing, clear watery snot, nasal itching, and nasal congestion, with symptoms lasting or accumulating for more than 1 h per day and (b) allergen testing: at least one allergen SPT and/or serum specific IgE positive; with a TNSS score [12] ≥ 4; and aged 18 to 65 years were included.

#### 2.2.2. Exclusion Criteria

Patients with acute sinusitis or respiratory tract infection within the last two weeks; with anatomical abnormalities such as deviated nasal septum, nasal stenosis, nasal polyps, acute and chronic sinusitis, nasal foreign bodies, or other occupying lesions; with a history of drug allergy; during pregnancy or lactation; and with severe lung, liver, or kidney disease or other serious primary diseases were excluded.

### 2.3. Treatment Methods

#### 2.3.1. Control Group

The patients in the control group received 10 mg of oral loratadine (Shanghai Schering-Plough Pharmaceutical Co., Ltd., State Drug Administration H10970410) daily at bedtime and 50 *μ* mometasone nasal spray (Zhejiang Xianju Pharmaceutical Co., Ltd, GMPZ H20113481) thrice daily in the morning, midday, and evening, respectively. A similar treatment regimen of loratadine and mometasone nasal spray was introduced to the patients in the study group.

#### 2.3.2. Study Group

The study group additionally received the Tuomin Zhiti decoction. The formula of the decoction is as follows: Fructus Mume 20 g, *Periostracum cicadae* 10 g, *Ganoderma lucidum* 10 g, Bulbus Lilii 20 g, Radix Scutellariae 10 g, Flos Magnoliae 10 g (wrapped with gauze when decocted), Fructus Xanthii 6 g, and *Radix saposhnikoviae* 12 g. Additional herbs were added according to patients' symptoms, 10 grams of *Radix angelicae Dahuricae* and 10 grams of mint for heavy nasal congestion and runny nose, 10 grams of Fructus Liquidambaris and 10 grams of Radix Stemonae for itchy nose and eyes, 20 grams of raw Radix Scutellariae, 15 grams of stirred fried *Rhizoma atractylodis Macrocephalae*, and 10 grams of *Radix saposhnikoviae* for allergy to cold air. The above herbs were decocted in water and administered in one dose a day, with a half dose in the morning and the other half in the evening. All decoctions were decocted by the pharmacy department of our hospital. The duration of treatment was 4 weeks.

### 2.4. Observation Indexes

#### 2.4.1. Clinical Efficacy

With references to guidelines for clinical research on new Chinese medicines, the clinical efficacy was divided into markedly effective, efficient, and ineffective according to the degree of alleviation of symptoms and the follow-up results of patients. Markedly effective: symptoms such as nasal congestion and runny nose disappeared and there was no recurrence in the follow-up. Effective: symptoms such as nasal congestion and runny nose were significantly alleviated, with occasional recurrence in the follow-up. Ineffective: No significant alleviation in symptoms such as nasal congestion and runny nose were observed, which required other treatment methods. Total efficacy = (markedly effective + effective)/total number of cases *∗* 100%.

#### 2.4.2. Nasal Symptom Scores

Total Nasal Symptoms Scores (TNSS) were used to assess patients' nasal symptoms, which were divided into 4 symptoms: nasal itching, sneezing, runny nose, and nasal congestion. The degree of symptoms was assessed by the patients: 0 for no symptoms, 1 for mild symptoms, 2 for moderate symptoms, and 3 for severe symptoms, with a total score of 12 points. The higher the score, the more severe the symptom [12].

#### 2.4.3. Quality of Life Score

The Rhinoconjunctivitis Quality of Life Questionnaire (RQLQ) [13] was used to assess patients' quality of life, including 28 questions in 7 domains (mobility, sleep, febrile symptoms, practical problems, nasal symptoms, ocular symptoms, and emotional aspects), with each item scored 0∼6 points, where 0 is no distress, 1 is slight distress, 2 is mild distress, 3 is moderate distress, 4 is severe distress, 5 is greatly severe distress, and 6 is extreme distress. The higher the score, the more severe the symptoms.

#### 2.4.4. Serological Indexes

Before and after treatment, fasting venous blood was collected from the patients, and serum interleukin 4 (IL-4) and interferon-*γ* (IFN-*γ*) were determined by enzyme-linked immunosorbent assay (ELISA).

#### 2.4.5. Eosinophil Count and Eosinophil Cationic Protein

Before and after treatment, the peripheral blood eosinophil count (EOS) was measured with an automatic blood cell analyzer, and eosinophil cationic protein (ECP) was measured by ELISA.

#### 2.4.6. Comparison of Follow-Up Results

After treatment, the patients were followed up for 12 weeks, and the incidence of nasal congestion, runny nose, and nasal itch was recorded every 2 weeks.

### 2.5. Statistical Analysis

SPSS 22.0 software was used for data analyses, and GraphPad Prism 9.0 was used to plot the graphics of the data. The count data are expressed as rates and analyzed using the chi-square test, and the measurement data are expressed as mean ± standard deviation ($\bar{x}\pm s$) and analyzed using the *t*-test. The Kaplan–Meier curve was used to analyze the recurrence. A statistically significant difference threshold was set at *α* = 0.05.

## 3. Results

### 3.1. Comparison of Baseline Data

As shown in Table 1, the comparison of baseline data such as age, gender, disease duration, smoking history, and sensitization status between the two groups of patients showed no statistically significant differences (all *P* > 0.05).

### 3.2. Comparison of Clinical Efficacy

As shown in Table 2, the control group had 14 cases of markedly effective, 18 cases of effective, and 18 cases of ineffective, with a total efficacy of 64% (32/50). The study group had 22 cases of markedly effective, 21 cases of effective, and 7 cases of ineffective, with a total efficacy of 86% (43/50). A significantly higher total efficacy was observed in the study group than that of the control group (*χ*2 = 6.453, *P*=0.006).

### 3.3. Comparison of TNSS and RQLQ Scores

As shown in Figure 1, there was no significant difference in the comparison of TNSS and RQLQ scores between the two groups before treatment (*P* > 0.05). The TNSS and RQLQ scores were significantly decreased after four weeks of treatment but without intergroup differences. Three months after treatment, the TNSS and RQLQ scores of patients in both groups rebounded significantly but were still lower than those before treatment, and the results of the study group were significantly lower than those of the control group (*P* > 0.01).

### 3.4. Comparison of Serum Inflammatory Factor Levels

As shown in Figure 2, there was no significant difference in IL-4 and IFN-*γ* between the two groups before treatment (all *P* > 0.05). After treatment, the two groups obtained remarkably decreased IL-4 levels and elevated IFN-*γ* levels, with better results being observed in the study group than in the control group (*P* > 0.001).

### 3.5. Comparison of Eosinophil Counts and Eosinophil Cationic Protein Levels

As displayed in Table 3, the two groups did not differ in terms of EOS and ECP before treatment (*P* > 0.05). After treatment, the two indicators showed a significant decline in both groups, in which the study group had lower results (*P* > 0.001).

### 3.6. Comparison of Follow-Up Results

Patients in both groups were followed up for 12 weeks after treatment, with no missed visits. As presented in Table 4, the recurrence rates at 6 and 12 weeks were 18% (9/50) and 56% (28/50) in the control group and 16% (8/50) and 28% (14/50) in the study group, respectively, with significant differences between the two groups absent in the 6-week recurrence rate (*P* > 0.05) and present in the 12-week recurrence rate (*P*=0.002). The recurrence curve was analyzed using the Kaplan–Meier method, HR = 2.251, 95% CI: 1.228 to 4.127 (*P*=0.007) (Figure 3).

## 4. Discussion

Allergic rhinitis is a chronic noninfectious inflammatory disease caused by the immune system on exposure to airborne allergens and is associated with symptoms such as nasal congestion, runny nose, sneezing, red itchy eyes with tearing, and swelling eyes [14]. AR seriously disrupts patients' daily life and may develop into allergic asthma and allergic conjunctivitis [15]. The treatment of AR includes four main aspects, namely, environmental management (allergen avoidance), pharmacotherapy, allergen-specific immunotherapy (desensitization therapy), and health education. The existing treatment and management are mainly used to relieve the symptoms and improve the quality of life of patients. Loratadine is a second-generation long-acting tricyclic antihistamine with a fast onset and strong effects. It is hormone-free and metabolized to more active desloratadine after human absorption, which inhibits histamine-induced allergic symptoms by competitively inhibiting histamine H1 receptors without significant anticholinergic and central inhibitory effects. Loratadine is widely used for the relief of AR-related symptoms such as sneezing, runny and itchy nose, ocular itching, and burning sensation [16]. Mometasone is a topical glucocorticoid and nasal spray administration exerts local anti-inflammatory effects at doses that do not provoke systemic effects [17]. The combination of loratadine and mometasone furoate has been investigated to be well tolerated and effective in controlling the symptoms of rhinitis [18].

In the present study, the total efficacy of the study group was significantly higher than that of the control group; after treatment, the study group obtained higher TNSS and RQLQ scores, better IL-4 and INF-*γ* levels, significantly lower levels of EOS and ECP, and a lower 12-week recurrence rate than the control group. The TNSS are the main index for the evaluation of the treatment efficacy of AR, RQLQ is the preferred scale to assess the quality of life of AR patients, IL-4 and INF-*γ* are the main factors to evaluate the inflammatory responses, and EOS and ECP are closely related to the severity of AR [19, 20]. The treatment of AR in TCM advocates the combination of physique identification with disease identification and evidence-based treatment, which enables rapid control of the disease, shortens the course of treatment, and reduces the dosage of Western medicine. The Tuomin Zhiti decoction is designed based on the idea of “key prescriptions for primary symptoms.” Symptoms such as nasal itching, sneezing, nasal runny nose, and nasal congestion are inherently triggered by the poor physique and the external invasion of evil qi, in which the poor physique refers to the allergic constitution and foreign qi invasion indicates the allergen. External cold or temperature changes may elicit or aggravate the disease, which occludes the skin and tissues and intensifies the fever and heat, thereby disturbing the nose [21]. The Tuomin Zhiti decoction stresses the treatment of both the physique and disease of the patients. *Periostracum cicadae*, Fructus Mume, and *Ganoderma lucidum* desensitize the body. Radix Scutellariae, *Periostracum cicadae*, Flos Magnoliae, Fructus Xanthii, and *Radix saposhnikoviae* dispel the evil and open the orifices, and the combination with Fructus Mume astringents the lung qi to prevent excessive dispersion of heat. The combination of the herbs desensitizes the body, clears the internal heat, and disperses the external evil. The decoction also emphasizes clearing and moistening. In the formula, Radix Scutellariae clears volatile heat and Bulbus Lilii nourishes Yin and eliminates dryness. This combination of clearing and moistening relieves the symptoms of a dry and itchy nose and prevents volatile heat from damaging Yin. Furthermore, the efficacy of the Tuomin Zhiti decoction also stems from its dispersal and astringency of qi. The composition of Flos Magnoliae, Fructus Xanthii, *Radix saposhnikoviae*, and Fructus Mume lowers the risk of excessive dispersion. In addition, an individualized treatment is provided through adjustment of the herbal medicines to achieve accurate treatment of symptoms [22]. However, there are still some limitations to this study. First, the application of TCM is adjusted according to symptoms in different patients, resulting in difficulties in the formulation of a unified plan for reference. Second, the present study is a single-center study with limited enrollments and follow-up, so the data may be insufficient to prove the efficacy in all patients. In future, a standardized treatment training and more prospective randomized controlled study will be carried out to provide more reliable data.

## 5. Conclusion

The Tuomin Zhiti decoction for the treatment of AR patients alleviates the clinical symptoms, reduces the inflammatory response, enhances immune function by regulating IL-4 and IFN-*γ*, and lowers the long-term recurrence rate.

## Figures and Tables

**Figure 1:** Comparison of the TNSS and RQLQ scores at different timepoints. TNSS = total nasal symptoms scores, RQLQ = rhino-conjunctivitis quality of life questionnaire, ^*∗∗*^ indicates *P* < 0.01and ^*∗∗∗*^ indicates *P* < 0.001.

**Figure 2:** Comparison of serum levels of IL-4 and IFN-*γ*. IL-4 indicates interleukin 4, IFN-*γ* indicates interferon-*γ*, ^*∗∗∗*^ indicates *P* < 0.001.

**Figure 3:** Comparison of the Kaplan–Meier curve of the recurrence rate.

**Table 1:** Comparison of the baseline data.

	Control group (*n* = 50)	Study group (*n* = 50)	*t*/*χ*2	*P*
Age (years)	34.56 ± 6.42	36.19 ± 7.03	1.211	0.229
Duration (years)	2.03 ± 0.51	1.98 ± 0.42	0.535	0.594
Gender			1.051	0.153
Male	33	28		
Female	17	22		
Smoking			1.004	0.158
Yes	29	24		
No	21	26		
Sensitization status			0.832	0.181
Monosensitized	15	11		
Polysensitized	35	39		

HDM = house dust mite.

**Table 2:** Comparison of the clinical efficacy.

	Markedly effective	Effective	Ineffective	Total efficacy
Control group (*n* = 50)	14	18	18	32 (63%)
Study group (*n* = 50)	22	21	7	43 (86%)
*χ*2				6.453
*P*				0.006

**Table 3:** Comparison of the EOS and ECP.

	EOS (%)		ECP (ng/L)	
	Before	After	Before	After
Control group (*n* = 50)	5.46 ± 1.32	1.56 ± 0.43	33.74 ± 6.73	17.78 ± 3.56
Study group (*n* = 50)	5.57 ± 1.41	1.14 ± 0.35	35.17 ± 7.03	14.36 ± 2.83
*t*	1.124	8.404	1.061	5.318
*P*	0.264	<0.001	0.291	<0.001

**Table 4:** Comparison of the recurrence rate in 6 weeks and 12 weeks.

	6 weeks recurrence rate	12 weeks recurrence rate
Control group (*n* = 50)	18% (9/50)	56% (28/50)
Study group (*n* = 50)	16% (8/50)	28% (14/50)
*χ*2	0.071	8.046
*P*	0.359	0.002

## Data Availability

The datasets used and analyzed during the current study are available from the corresponding author on reasonable request.
